RETRACTED

# Preparation of PCL Electrospun Fibers Loaded with Cisplatin and Their Potential Application for the Treatment of Prostate Cancer

**DOI:** 10.1155/2022/6449607

**Published:** 2022-07-15

**Authors:** Hilla Mills, Ronald Acquah, Nova Tang, Luke Cheung, Susanne Klenk, Ronald Glassen, Magali Pirson, Alain Albert, Duong Trinh Hoang, Thang Nguyen Van

**Affiliations:** ^1^Department of Medical Science, University for Development, Accra, Ghana; ^2^RD Lab, The Hospital Institute for Hebal Research, 50200 Toluca, Mexico, Mexico; ^3^Research Institution of Clinical Biomedicine, Hospital University Medical Centre, 89000 Ulm, Germany; ^4^Industrial Research Group, International College of Science and Technology, Route de Lennik 800, CP 590, 1070 Brussels, Belgium; ^5^Clinical Analysis Lab, Center of Bio-Medicine, Hanoi, Vietnam

## Abstract

Prostate cancer is a global fatal type of cancer. It is a type of cancer that affect men. Signs and symptoms of the disease include blood in the urine, pain when one micturates, and difficulties in penis erection. Cisplatin chemotherapy is a principal treatment normally given to the prostate cancer patients. Nonetheless, on its own, cisplatin loses efficacy once administered due to liver pass effects and other biochemical attacks. In this paper, we looked at preparation of PCL nanoparticles loaded with cisplatin and their potential for the treatment of prostate cancer. PCL nanoparticles protect cisplatin from biochemical attack, thus increasing drug efficacy. Incorporation of P-glycoprotein inhibitors in PCL nanoparticles (NPs) loaded with cisplatin could improve prostate cancer treatment even more.

## 1. Cisplatin

It is reported that Rosenberg and colleagues unintentionally observed that cisplatin (Figure 1) has cytotoxicity effects characterized by high antitumor activities. The observation dates back to 1960s. Approximately a decade down the line, cisplatin became the world-renown first platinum-based cancer drug in the medical field. Cisplatin was first introduced by Michele Peyrone in 1845 as a platinum-based chemotherapy [1]. Thereafter, it became the drug for the treatment of majority of cancers, namely, lung cancer, ovarian cancer, testicular, head and neck malignancies, among others. Cisplatin was then modified to give a variety of platinum-based drugs, which were also anti-cancer agents. These cisplatin analogues include nedaplatin, oxaliplatin, and carboplatin [1–3]. Notwithstanding this, cisplatin and its analogues were used limitedly owing to their cross-resistance, toxicity, and poor solubility [4]. These factors were then improved by the development of nanotechnology [5].

Norio Taniguchi is given a credit for coming up with a term nanotechnology in 1974. He defined nanotechnology as the capability to engineer materials of magnitude 10^−9^ m precisely. The modern definition of nanotechnology is the design and “tailor-making” of devices, materials, and systems with control at nanometer dimensions. According to Jeremy [6], a distinction is made between nanoscience and nanotechnology. Nanoscience focuses on the study and observation of “events” at the nanometer scale. In addition, nanoscience involves the ways of manipulating matter at that scale. The discrepancy between the two terms is of no great significance; nonetheless, nanotechnology is versatile. Physics, chemistry, biology, and medicine, among others, are fields where nanotechnology is of great importance.

RETRACTED

A thorough study of platinum-derived anti-cancer drugs was feasible due to a rapid nanotechnology development [7]. During the preparation or synthesis of cisplatin and its analogues, *cis*-diamminediiodoplatinum (*cis*-DIDP) is the intermediate compound. Both cisplatin and *cis*-DIDP are square planar complexes. The only difference is that chloride ions are substituted by iodide ions in *cis*-DIDP. Cisplatin is less unstable than *cis*-DIDP according to the spectrochemical sequence of crystal field theory. Consequently, iodide ion is a better leaving group than the chloride ion in an aqueous environment [8, 9]. One, therefore, can see that *cis*-DIDP is more of an anti-cancer drug than an intermediate. A number of methods can be employed to enhance therapeutic indices of platinum-derived anti-cancer drugs. Examples of such methods are preparation of drug carriers like polymers, polymeric micelle, cancer-targeting formulations of platinum-containing drugs development, and long-circulating liposome [10–12]. Once controlled-release drug carriers are well developed, cis-DIDP can be an excellent anti-cancer drug [5].

## 2. Electrospinning

Electrospinning can also be referred to as electrostatic spinning. The formation of micro/nano-sized polymeric fibers either solid or hollow by the applying an electric force on the polymeric solution at the sharp end of a conducting tube is referred to as electrostatic spinning [13–15]. The technique had been highly used for the past 30 years, and its application is still elevating. In 1745, Bose and colleagues became pioneers to describe the formation of aerosols by applying an electric potential to the fluids [16]. It is reported that Lord Rayleigh went on to quantify the charge required by the fluid to surmount the surface tension of a drop. Morton and Cooley designed and made a first device to spray liquids under the influence of electric charge. The duo patented the device in 1902 and 1903. Kiyohiko fabricated artificial silk in 1929 [16]. During the time spun from 1940 to 1960, studies were confined to obtaining uniform-sized particles, designing the instruments, decreasing the size, and understanding and optimizing parameters [17, 18]. It is reported that, by 1990 onwards, fabrication process was incorporated in the curriculum of many educational institutions. A lot of studies, since then, have been conducted on the applications and versatile production of the electrospun-particles [19].

RETRACTED

### 2.1. Process

The electrostatic spinning process requires a high voltage supply of either negative or positive polarity to charge the polymer solution, a syringe, a syringe pump, and a grounded collector. It is recommended that electrospinning procedures are carried out in a hood with minimum atmospheric pressure. The precaution serves to protect both personnel and fibers according to [19]. Upon the accumulation of sufficient repulsive force and a phenomenon when the repulsive force counterbalances the surface tension, on the conducting tube, the drop surface begins to form what is referred to as the Taylor cone. It is reported that, at an angle of 49.3°, the conducting polymer solution can reach an equilibrium state where it forms a cone in an electric field [20]. Further, increments in the electric field strength result in the repulsive force outpowering the surface tension. Consequently, liquid jet formation from the Taylor cone occurs due to sufficient intermolecular and intramolecular forces in the solution. In an event that there is no suffice force of attraction or cohesive attraction, the jets break, and the particles formed are sprayed onto a collector plate. The fiber that originates from the Taylor cone moves through the air approaching the collector plate, and at the same time, the solvent vaporizes, forming solid fiber deposit onto the collector [18, 20]. The jet begins to be unstable for a short displacement following its voyage in the air and then begins to whip. As a result, a path to the collector plate is increased. The phenomenon helps in solvent vaporization and fiber thinning [19].

### 2.2. Electrospinning Physics

A gradual increase in electric field strength makes the drop surface to be convex-shaped at a particular voltage called critical voltage, *V*_c_. Once *V*_c_ is reached, sprays (electrospraying) and jets (electrospinning) begin to occur and can be modelled by the following equation:

(1) $$\begin{array}{c} Vc=\frac{H^{2}}{L^{2}}\left(Ln\frac{2L}{R}-\frac{3}{2}\right)\left[0.117\pi \gamma R\right]. \end{array}$$

The parameters are defined as follows: H is the distance between the capillary and the collector; *γ* is the surface tension; and R is the radius of the capillary [20]. Hendrick and colleagues came up with an equation that relates potential (V) to *γ* and *r* (radius of the pendant drop). The potential (V) that is needed for electrospraying a charged pendant polymer drop solution from that in capillary is computed using the following equation:

(2) $$\begin{array}{c} V=300\sqrt{\left(20\pi \gamma r\right)}. \end{array}$$

[21].

RETRACTED

Two important parameters, namely, viscosity and conductivity, are not included in the equation modelled by Hendrick and colleagues regardless the fact that they are crucial electrospinning parameters. Equation (1) is valid for sparingly conducting medium to low conducting solutions [19].

## 3. Electrospinning Parameters

Electrospinning is a simple technique. Howbeit, solution parameters, and process parameters affect uniformity, porosity, and size of fibers. Studies have been done to try and grasp these parameters; notwithstanding this, the parameters are not universal. Different modifications in any of the parameters by different researchers in a certain polymer yield different results with another polymer. Below are the crucial parameters to be considered [19].

### 3.1. Voltage

The voltage supply is one of the principal factors that affect production of fibers. The electric filed strength matters. Formation of jet, beads, and the size of the fiber all depend on the voltage supplied. If one increases the voltage of a polyethylene oxide (PEO)/water system, the site at which the jet originates changes from the tip of the pendant drop to the tip of a capillary. Simultaneously, pendant drop volume decreases [18, 22]. One ought to bear in mind that the jet experiences instability right from the onset of the electrospinning process. Reduction in the electric field strength shifts the position of instability towards the tip of the capillary [23]. Chun and Reneker observed an insignificant fiber diameter change with a change in voltage supply when working with PEO solution [24]. Megelski and colleagues reported that polystyrene fiber size increased when the voltage supply was reduced. However, the team observed an insignificant change in the fiber pore formation [25]. Above 10 kV, electrospun polyvinyl alcohol (PVA)/water solution showed a variety of diameter distribution [26, 27]. The charge carried by the fibers to the plate serves to complete the circuit. As a result, there is a flow of current associated with electrostatic spinning process. When three parameters, namely, flow rate, dielectric constant, and conductivity, are kept constant, an increase in the current flow is noted, which means that the mass of fibers formed has increased. A small increment in current is noted from the beginning of the electrospinning process, and then a sharp increase is observed later from one voltage point. During electrospraying, things are different. Sharp increments in current are observed. Changes in bead density may explain the phenomenon of sharp change in current [19].

RETRACTED

Scientist wanted to know what happens if polarity is reversed. However, the findings were inconsistent. Kilic and colleagues carried out an experiment using 7.5 wt (%) PVA/water solution with an intention to study how production and morphologies of nanofibers respond to polarity reversal. The team inferred that a decrease in nanofiber production was because of destitute-columbic force on the jet. However, pore size and diameter of the web layer were found to be much finer and more evenly distributed [28]. Contrary to Kilic and colleagues' findings, Varesano et al. documented good quality production of nanofibers with multijet electrostatic spinning for both reverse polarity and conventional [29].

### 3.2. Rate of Flow

The rate at which the polymer solution flows has a direct effect on the porosity, shape, and size of fibers. According to Megelski et al., the diameter and pore size of fibers increased at a low flow rate. High flow rates caused bead defects [25]. These findings were for a polystyrene/tetrahydrofuran (THF) solution. Similar morphological effects were reported in a different study using 20 wt (%) nylon-6-formic acid solution at different flow rates at a constant electric field strength of 20 kV. A noble Taylor cone and narrowest fiber diameter distribution were observed at a flow rate of 0.5 ml/h. Notwithstanding this, at a flow rate of 0.1 ml/h, the team observed that the Taylor cone could not be maintained. It could not be reduced with time in order to obtain fiber from within the capillary tips It was observed that, for 1.0 and 1.5 ml/h flow rates, the electric field could not suffice to spin all the solution. Few drops were sprayed, breaking off from the capillary because of the force of gravity [19].

### 3.3. Distance between Capillary and Collector

According to Bhardwaj and Kundu [30], the capillary-collection distance affects the shape and size of nanofibers. Careful adjustments need to be done with an intention to achieve optimum capillary-collector distance, which allows the production of quality fibers. It is believed that this factor (capillary-collector distance) could be the key parameter that contrasts electrospraying and electrospinning. Nurwaha et al. [31] asserted that a capillary-collector distance that falls within a range of 10–20 cm is effective when one uses the conventional method of electrospinning. The large distance from the Taylor cone had an effect of decreasing the fiber diameter [32]. Similar observations were reported by Jaeger and colleagues. Distance increments from 1, 2 to 3.5 cm changed the diameter of the fiber from 19, 11 to 9 *μ*m, respectively. The distance was measured from the capillary orifice to the collector [23].

RETRACTED

### 3.4. Solution Concentration

Surface tension and viscosity of the polymer solution are the two crucial parameters that cannot be ignored when it comes to the electrospinning process. It recorded that surface tension outweighs viscosity in a low concentration solution. In such a solution, it is difficult to form continuous fibers; instead, drops will be formed. Solutions of this nature are said to have viscosity, which is less than 1 poise. Highly concentrated solutions of viscosity greater than 20 poise are difficult to maintain when they start to flow. According to a statistical study conducted by Sukigara et al. on regenerated silk, silk concentration proved to be the crucial parameter in producing uniformity in fibers of less than 100 nm [33]. Another study by Fong and colleagues on PEO solutions with an intention to understand the effects of viscosity on bead formation is worthy to consider. The team observed that solution viscosity did affect not only bead density, but also bead diameter. A bead morphological change from spherical to spindle-like fibers was observed at higher viscosities [21]. In addition to that, high surface tension-low concentration polymer solutions produced droplets due to insufficient viscoelastic forces to surmount charge repulsive forces. Viscoelastic forces at higher concentrations are large enough to prevent the formation of fiber fragments, thus forming smooth nanofibers [34].

### 3.5. Viscosity

Fiber formation is governed by solution viscosity. One can obtain smooth continuous fibers at optimum viscosity for a certain polymer solvent combination. Factors like concentration, viscosity, and molecular weight of a particular polymer solution are related, and thus, it is not easy to look at them separately in an effective manner. High electric filed strengths required at high viscosity and thus difficult to manage [33, 35]. According to Baumgarten [34], droplets that were formed at low viscosity were not completely dry. Droplets collided with each other in mid-air because of incomplete drying at higher viscosities with acrylic polymer. A solution mixture of dimethylformamide (DMF) and ethanol in the ratio 50 : 50 was suggested by Yang et al. for obtaining best poly(vinyl pyrrolidone) electrospun fibers [36].

### 3.6. Molecular Weight

Polymer molecular weight influences polymer solution viscosity. Consequently, a relationship between polymer molecular weight and viscosity is crucial, as it determines fiber morphology. When one decreases the PVA molecular weight and keeps all other parameters constant, bead-like structures are formed. Higher molecular weight results in the formation of smooth fibers at the beginning of the process than ribbon-like structures on further increments in molecular weight [37]. According to Zhao et al. [38], ultra-high molecular weight polymers like polyacrylamide showed a broad spectrum of morphologies even when small changes in concentration were made within the range of 0.3–3.0 wt (%). Smooth and bead-like fibers formed within 0.3–0.7 wt (%) concentration range. At higher concentration range (0.7–2.0 wt%), both ribbon-like and smooth fibers coexisted. Above 2.0 wt (%), helical ribbon-like structures or zig zag ribbons with triangular beads on them were formed. The experiment on melts polypropylene revealed a linear relationship between molecular weight and fiber diameter. A very high degree of entanglement was noted in high-molecular weight polymers and thus daunting for electric filed to pull on each and every polymer chains so as to obtain a thin fiber [39].

RETRACTED

### 3.7. Surface Tension

Molecules possess forces that hold them together. In solutions, such forces are called cohesive forces and are responsible for the surface tension. Surface tension depends on solvent, polymer, and the solution composition. A study conducted by Yang et al. on the effect of solvents on nanofiber formation using poly(vinyl pyrrolidone) revealed that high viscosity with lower surface tension solvent properties of ethanol produced smooth nanofibers. The team recommended the use of multisolvent system in order to obtain optimum viscosity and surface tension for better fiber qualities [36]. Surface tension determines the types of solvents and their concentrations that are required for the electrospinning process [26].

### 3.8. Surface Charge Density and Conductivity

The surface charge density of polymer solution and conductivity play a critical role during the electrostatic spinning process. High conductivity polymer solutions carry great charge. Highly conductive solution experiences stronger tensile force in the electric field and is thus conducive to electrospinning. The diameter of the nanofibers significantly decreases with the increase in solution conductivity. The relationship can be simplified by stating that the radius of the fiber jet is inversely proportional to the cube root of solution conductivity [40]. According to Baumgarten [34], jet radius is dependent on the reciprocal of the electrical conductivity cube root for acrylic microfiber preparation. Natural polymers are polyelectrolytic and possess a better charge-carrying capacity than synthetic polymers. However, synthetic polymers form better fibers than natural polymers [41]. According to a study conducted by Hayat and colleagues, semiconducting liquid produced stable jets when sufficient voltage was applied. Solvents like paraffin oil could not built a surface electrostatic charge because of insufficient free charges, whereas water produced sparks at higher voltage supplies and unstable stream. Therefore, semiconducting and insulating liquids could produce stability in fibers [42]. A different study on PVA solution revealed that, upon addition of minute amounts of sodium chloride, solution conductivity increased sharply and yet decreasing the fiber diameter at the same time [27]. Frequency of beads formation decreased upon the addition of sodium chloride in PEO solution [21]. Compounds like lithium bromide, ammonium chloride, potassium phosphate, and sodium phosphate can be used to improve fibers by changing solution conductivity [21, 41]. Huang and colleagues used organic-solvent-soluble compounds like pyridine that react in solution with formic acid to form a salt. Pyridine does not only improve conductivity, but the fact that it is not difficult to remove so that dry fibers are obtained makes it favorable. According to Huang et al. [17], adding 0.4 wt (%) pyridine had an effect of doubling the electrical conductivity of 2% nylon-6-formic acid [19].

RETRACTED

### 3.9. Solvent Volatility

It is reported that the time taken by the jet from the capillary orifice to the collector might be fewfold more than the capillary-collector distance. Dry, porous fibers are formed during electrospinning depending on the choice of solvent to solubilize the polymer. If a scenario that the fibers do not completely dry occurs, the fibers attach themselves in the mid-air forming ribbon-like fibers [25]. If the phenomenon does not occur in the mid-air, it occurs on the collector. A research that was done on polystyrene fibers exhibited that a more volatile tetrahydrofuran (THF) solvent did not only produce high-density pores, but also increase the fiber surface area by up to 40%. Nonetheless, the same polymer in DMF completely lost the macrotexture. Different morphological profiles were obtained when THF-DMF solvent mixture ratios were varied [19].

## 4. Nanofibers as Drug Delivery Agents

Regardless the prominence of nanotechnology in drug delivery process, one ought to grasp conditions on the technology that is of maximal benefit. According to Sill and von Recum [18], for drug delivery, the materials used should be biodegradable and biocompatible, respond to stimuli, possess mass transfer properties, and permit drug loading, only to mention a few.  Table 1 highlights some of the advantages and disadvantages of nanofibers as drug-carrying agents.

RETRACTED

### 4.1. Material Used for Nanofiber Production

A broad spectrum of polymers has been used for the production of nanofibers. Such polymers include poly(L-lactide-co-caprolactone), poly(ethylene oxide), poly(*ɛ*-caprolactone), poly(lactic acid), poly(D,L-lactide-co-glycolide), poly(ethylene glycol), poly(urethane), poly(carbonate), poly(caprolactone), poly(glycolic acid), and poly(L-lactic acid). Nonetheless, not all of them are used for drug delivery purposes [45].  Table 2 shows the examples of materials used for drug delivery.

### 4.2. Poly(*ɛ*-Caprolactone)

Poly(*ɛ*-caprolactone) (PCL) is a bioresorbable, biocompatible, and biodegradable polymer. It belongs to the aliphatic polyester family. The aliphatic polyester family has many applications in many areas. It is of great importance in drug delivery systems, fixation devices, contraceptive devices, and wound dressing [48]. PCL is well known when it comes to drug delivery aspects. Notwithstanding this, PCL is not limited to that area; rather, its use has been extended to vaccines, peptides, proteins, and other bioactive molecules. Preparation of PCL mainly involves polymerization process using a monomer and an initiator. A monomer and an initiator are mixed at high pressures under purging nitrogen, thus resulting in polymer formation. The obtained polymer is allowed to cool. Afterwards, the polymer is dissolved in an organic solvent and then washed to get rid of remaining unreacted molecules. Freeze-drying the resultant polymer is necessary as a way of preserving the polymer for future use [49].

### 4.3. Synthesis

Two different methods can be used to synthesize PCL namely ring opening polymerization (ROP) of *ɛ*-caprolactone [50] and polycondensation of 6-hydroxyhexanoic acid. Polycondensation involves a step-by-step series of chemical reactions. Two molecules of complementary nature in terms of functional groups react allowing chain elongation and releasing small molecules. The acidic functional group of 6-hydroxyhexanoic acid or that of a growing polymer chain reacts with the hydroxyl group of another 6-hydroxyhexanoic acid. Water molecules are produced during this esterification reaction, in addition to the growing polymer chain. Water production during the synthesis of PCL is crucial since it enhances the equilibrium to favor the products side [51]. Polycondensation, however, is not a favorable method for PCL synthesis. A better method for PCL synthesis is the ROP because polymers with lower polydispersity values and higher molecular weight are attainable. The method comes in different versions, namely, monomer-activated, coordination insertion, and anionic and cationic ROP. Generally, the ROP process is a solution or bulk process in which a polymeric chain that possesses a propagating center allows the addition of cyclic monomers to the structure. The ring strain drives the process. Initial monomer concentration and temperature are crucial when it comes to morphologies of the products [49].

RETRACTED

### 4.4. PCL Physicochemical Properties

Polycaprolactone has the melting temperature, which falls in the range of 332–337 K. The melting temperature depends on the crystallinity of the subject polymer. PCL blends well with other polymers, and its melting temperature enhances scaffold formation. The polymer's glass transition temperature is 213 K. The heat of fusion of a pure (100%) crystalline PCL is 139.5 kJ/kg, which can be used as a crystalline standard to estimate crystalline level of PCL. One good property of PCL is its solubility in a number of solvents [52].

### 4.5. Methods of Incorporating Drugs Using Electrospinning Process

Electrohydrodynamic (EHD) technology allows the formation of nanofibers with a broad spectrum of morphologies and sizes. Different techniques like surface modulation, coaxial, emulsion, electrospray, and blending, among others, are employed to incorporate drugs and bioactive molecules like DNA and growth factors. Each technique suits the nature of treatment desired [45].

### 4.6. Prostate Cancer

Prostrate affects the male reproductive system and is the second most prevalent cancer across the globe. It is reported that this type of cancer accounts for 10% of all cancers in males [53, 54]. According to Wilkinson and Chodak [55] and Wang et al. [56], prostate cancer incidences have increased significantly in China. Cisplatin chemotherapy is a principal method of prostate cancer [57]. However, the majority of chemotherapy drugs pose adverse effects even at therapeutic doses. Consequently, it is imperative to probe alternative effective therapeutic methods that may surmount drug toxicity [58].

### 4.7. Nanoparticles

Polymeric nanoparticles (NPs) are advantageous when it comes to drug delivery. They render drug stability. In addition, NPs reduce the cases of multidrug resistance (MDR), which is a very common phenomenon with other anti-cancer drugs. The mechanism by which polymeric NPs mitigate MDR is the ability of internalizing the drug, hence shielding it from efflux pumps like P-glycoprotein in cancer cells. It is reported that gold NPs have a higher affinity for cancer cells than normal mesenchymal cells; thus, gold NPs preferably destroy cancer cells. Regarding poly(lactic-co-glycolic acid) (PLGA) NPs, regardless their attractive attributes in drug delivery applications, a number of challenges have been encountered. It is daunting to target the diseased tissue using PLGA NPs. Also, a single polymer cannot escape the reticuloendothelial system. Some PLGA NP modifications can meet the aforementioned problems. The introduction biomimetic ligands and the biomolecular processes can reduce the challenges that come with PLGA NPs [59].

RETRACTED

### 4.8. Cisplatin Mode of Action

Platinum-based drugs destroy cancer cells by interrupting transcription. The formation of platinum-DNA adducts inhibits cancer cells division. The inhibitory effect of cisplatin is corrected with cancer cell deformation. The cancer cells shrink. The platinum-DNA adducts lead to programmed cell death. Cisplatin loses one of its chloride ligands and binds the DNA forming intrastrand DNA adducts. Consequently, nucleic excision repair (NER) mechanism is activated to try and tackle the DNA damage caused by the cisplatin. The NER is switched on by an activation of ataxia-telangiectasia mutated (ATM) pathway. Cisplatin-DNA adducts switch on a number of signal transduction that prevent programmed cell death. Recent studies revealed that p53 gene is associated with DNA damage and repair [46]. The tumor suppressor gene, p53, is maintained and phosphorylated by the activated ATM pathway. Consequently, transactivation of many genes like Bax, which facilitate apoptosis, DNA damage inducible gene 45 (GADD45), which takes part in DNA repair, and p21 gene, which arrests cell cycle growth, might be induced. The p53 gene helps in cisplatin-mediated apoptosis by binding to the Bax-xL directly, thus negating its antiapoptotic nature. Subsequently, the effectiveness of FLICE-like inhibitory protein (FLIP) needed for p53 gene to activate cisplatin-mediated apoptosis is decreased. The intrastrand lesions caused by cisplatin-induced DNA crosslinks activate the mismatch repair (MMR) system, which is known for potentiating tyrosine kinase c-Abl in response to stress caused by DNA-damaging agents. Extracellular signals that maintain cell growth and sustenance such as JNK and p38 mitogen-activated protein kinase (MAPK) are activated once the c-Abl is activated, to sustain tumor protein p73 resulting in programmed cell death [60].

## 5. Conclusions

Nanoparticles loaded with drugs for treatment of a broad spectrum of ailments are much more efficient than normal administration of “naked drugs.” A body consists of many barriers, namely, cell membrane, BBB, and so on. Barriers are not only a challenge, but also pumps and specialized enzymes that get rid of xenobiotics. Cytochrome P450 (CYP 450) enzymes, conjugating enzymes like glutathione, and liver pass effect account for decrease in drug efficacy. Cancer cells have a specialized pump known as P-glycoprotein, which render cancer cells resistivity to a number of anti-cancer agents like methotrexate, cisplatin, and many more. PCL/gelatin nanoparticles loaded with cisplatin increase the drug efficacy in treating prostate cancer since it shields cisplatin from attack by CYP 450 enzymes, gastric acid, glutathione, and many other proteins that get rid of xenobiotics, thus alleviating MDR. Loading cisplatin and P-glycoprotein inhibitor together in PCL nanoparticles could escalate the rate at which prostate cancer cells die, thus improving efficacy. A number of ways by which the PCL nanoparticles enter the targeted cells were reported. One of the major ways is receptor-mediated endocytosis. Once in the cell, the cytotoxic cisplatin mechanism is carried out to destroy cancer cells. Thorough understanding of electrospinning techniques and preparation of PCL and PCL nanoparticles loaded with cisplatin will significantly alleviate prostate cancer chaos globally [2, 8, 43, 60–62].

RETRACTED

## Figures and Tables

**Figure 1:** Cisplatin.

**Table 1:** Advantages and disadvantages of nanofibers as drug-carrying agents [43, 44].

Advantages	Disadvantages
High surface-to-volume ratio accelerates drug solubility in the aqueous environment and improves drug efficiency.	Scaffolds of nanofibers might be used as templates for the formation of conductive drug-loaded polymer systems.
Surface structure and morphologies of nanofibers make it possible to curb the drug dose and the rate at which the drug is released.	Production of nanofibers requires the use of organic solvents and it is impossible to control the 3-dimensional pore structure.
Bioactivity of the drug is maintained because biodegradable polymers shield the drug from corrosive attack by enzymes and gastric acid.	

**Table 2:** Examples of materials used for drug delivery [43, 46, 47].

Nanofiber	Drug(s) loaded	Drug properties
Poly (D,L-lactide-co-glycolide), PLGA/gelatin	Fenbufen	NSAID (non-steroidal anti-inflammatory drug).
PVA	Sodium salicylate, indomethacin, naproxen, and diclofenac sodium	Soluble, soluble, sparingly soluble and insoluble in water, respectively.
Poly (*ɛ*-caprolactone)	Naproxen	NSAID that belongs to the propionic acid. relieves fever, pain and swelling.
